The article "Study on the molecular mechanism of nightshade in the treatment of colon cancer" was retracted in 2023. Reasons: original data or images not available; unreliable results or conclusions; concerns about the data; concerns about the results or conclusions.

# Study on the molecular mechanism of nightshade in the treatment of colon cancer

**DOI:** 10.1080/21655979.2021.2016045

**Published:** 2022-01-11

**Authors:** Song Na, Li Ying, Cheng Jun, Xiong Ya, Zhang Suifeng, He Yuxi, Wang Jing, Lai Zonglang, Yang Xiaojun, Wu Yue

**Affiliations:** a Department of Oncology, Chongqing Traditional Chinese Medicine Hospital, Chongqing, 400020, China; b Department of Nephrology, Chongqing Hospital Of Traditional Chinese Medicine, Chongqing, 400020 China; c Department of Plastic and Cosmetic Surgery, Xinqiao Hospital, Army Medical University, Chongqing 400037, China; d Department of Gastroenterology, Chongqing Traditional Chinese Medicine Hospital, Chongqing, 400020, China

**Keywords:** Colon cancer, network pharmacological analysis, nightshade, quercetin

## Abstract

The present study attempts to explore the effective components, action targets, and potential mechanism of nightshade for colon cancer treatment. The relationship network diagram of ‘traditional Chinese medicine – component – target – disease’ was firstly constructed by employing network pharmacology. Experiments were conducted in vivo and in vitro to verify the influence of quercetin, the core effective component of nightshade, on colon cancer. Meanwhile, the regulatory effects of quercetin on core targets and main signaling pathways were determined. Based on the network diagram of ‘traditional Chinese medicine – component – target – disease’ and KEGG analysis, quercetin might exhibit certain effects on colon cancer treatment by regulating the biological behavior of core targets related to cell apoptosis in tumors including PIK3R1, PIK3CA, Akt1, and Akt2. Furthermore, quercetin has been demonstrated in vitro experiments to suppress the proliferation and migration of colon cancer cells whereas promote their apoptosis in a dose-dependent fashion. In vivo experiments indicate that quercetin had an antitumor effect on human colon cancer SW480 cells in nude mice bearing tumors. Furthermore, PIK3CA could bind to quercetin directly, which is validated by immunocoprecipitation. Therefore, the activation of PI3K/AKT phosphorylation was inhibited by quercetin and moreover the expressions of apoptotic proteins caspase-3 and Bcl2-Associated X protein (BAX) were up-regulated. In conclusion, the potential mechanism of nightshade lies in the activation of the PI3K/AKT signaling pathway inhibited by quercetin, thus promoting apoptosis of colon cancer cells for colon cancer treatment.

## Introduction

Colorectal cancer (CRC) is a frequently encountered gastrointestinal malignancy in clinical practice and responsible for approximately 930,000 deaths according to the global cancer statistics 2020 reported by the International Agency. It ranks the second place of most deadly cancers globally followed by lung cancer and fifth in China with 280,000 deaths. The results of disease screening have suggested that the incidence of CRC ranks the third worldwide and the second in China [1]. The current mainstream therapeutic options of CRC include surgery, radiotherapy, chemotherapy, and targeted therapy, whereas unsatisfactory efficacy and the key factor of death were resulted due to the occurrence of CRC invasion and metastasis at middle and advanced stages [2]. As early diagnosis and new drugs advance over the past decade, the average survival time of advanced CRC patients has doubled. Unfortunately, their survival rates remain low, typically the death occurs within 3 years [3]. Therefore, safe and effective medications in inhibiting tumor cell invasion and metastasis is a topic of trending and a challenge in the current research.

The article "Study on the molecular mechanism of nightshade in the treatment of colon cancer" was retracted in 2023. Reasons: original data or images not available; unreliable results or conclusions; concerns about the data; concerns about the results or conclusions.

Traditional Chinese medicine (TCM) boasts a long history of over 2000 years in the treatment of tumors. Based on the principle ‘treatment must rely on the causal root’, TCM diagnoses and treats patients in differentiation and benefits patients with malignant tumors in a favorable manner. Nightshade is the whole grass of *Solanum nigrum L*. in the *Solanaceae*. Modern studies have found that nightshade produces an anti-tumor effect and it has been extensively employed in treating multiple tumors [4]. Existing research results have shown that the anti-tumor mechanisms of nightshade mainly include blockage of the cell cycle, inhibition of cell proliferation and tumor growth, induction of cell apoptosis, and inhibition of epithelial-mesenchymal transformation and tumor metastasis [5], thereby enhancing the efficacy of radiotherapy, chemotherapy, targeted therapy, and reversal of drug resistance. Literature retrieval results have indicated that multiple active ingredients of nightshade contain solanine, solamargine, solaoiacid, solasonine, α-solanine, solasodine, degalactotigonin, quercetin, and diosgenin, can produce anti-tumor activities [6]. Experiments have revealed that solamargine mediates the proliferation of human colon cancer cell HCT-116 and enhances the activity of caspase-3 [7]. Quercetin can improve the radiotherapy effect of drugs in colon cancer, and the mechanism may link to the decrease of Notch-1 protein expression [8]. In recent years, an internationally recognized concept is prone to introduce multi-target drugs to treat complicated diseases. TCM has gained increasing concerns in the international medical community and drug discovery field owing to its multi-component and multi-target characteristics. The systematic and integrated research concept of network pharmacology coincides with the multi-components, multi-efficacy, and synergistic actions of TCM compounds. Currently, network pharmacology has achieved satisfactory results in the pharmacological mechanism of TCM [9]. Multiple studies have proved that network pharmacological analysis can be used as a technique of predicting active components and key targets of TCM for tumor treatment [10].

The article "Study on the molecular mechanism of nightshade in the treatment of colon cancer" was retracted in 2023. Reasons: original data or images not available; unreliable results or conclusions; concerns about the data; concerns about the results or conclusions.

Phosphatidylinositol 3-kinase (PI3K)/protein kinase B (PKB/Akt) signaling pathway produces an essential role in tumorigenesis, development, and radiation resistance [11]. It is involved in several cell activities and metabolism regulation and is intimately correlated with cancer cell proliferation and apoptosis, cycle regulation, angiogenesis, invasion, metastasis, and chemoradiotherapy resistance [12,13]. Moreover, Fei Zhou et al. found that resistance could be exacerbated in colon adenocarcinoma via activation of the PI3K/AKT signaling pathway [14]. It is therefore that targeted therapy for the important targets of the PI3K signal transduction pathway turns into a hot research topic for most researchers. More targeted inhibitors have been discovered with satisfactory effects. Several studies have proposed that multiple natural active ingredients play an anti-tumor role through targeting PI3K/Akt signaling pathway.

Taken together, this work initially screened the active components and action targets of nightshade on a network pharmacological approach with the hypothesis of the main component quercetin exhibiting as effective element in treating colon cancer. We designed several cell experiments aiming at examining whether quercetin affected the viability, apoptosis, migration, and invasion of tumor cells. A nude mouse model of tumorigenesis was employed to assess whether quercetin produces any effects on the mice, and relevant molecular mechanism of quercetin anti-tumor was explored using a molecular experimental technique to provide a basis for the application of the TCM nightshade in treating colon cancer.

## Materials and methods

### Network pharmacological analysis

In light of the pharmacokinetic characteristics of the components, the screening criteria were set as oral bioavailability (OB) ≥ 30% and drug likeness (DL) ≥ 0.18 [15], and TCM components, the main active components of nightshade were obtained from Traditional Chinese Medicine Systems Pharmacology Database and Analysis Platform (TCMSP, https://tcmsp-e.com/) database [16]. Then, structures of Canonical SMILES strings of the obtained active ingredients were collected through the PubChem database [17], imported into the Swiss Target Prediction database [18] and targets of active ingredients were downloaded, those with the probability > 0 were selected. Keywords colorectal cancer were input into the GeneCards database [19] (http://www.GeneCards.org/) and genes of relevance score > 10 were exported and collected as gene targets of colon cancer. The Venn diagram was plotted to obtain the overlapped targets of the disease and the herb [20]. The previously described data of the drug, active components, overlapped targets, and disease were imported into the Cytoscape 3.7.2 software. The corresponding diagram was generated subsequently. Nodes of different shapes represented the drug, active components, corresponding targets, and disease. Connecting lines represented the relationship between different components. Finally, ClueGo, a plugin for gene ontology (GO) enrichment analysis and Kyoto Encyclopedia of Genes and Genomes (KEGG) pathway enrichment analysis for the overlapped targets [21,22], and the 20 pathways with the highest P values were sorted out.

The article "Study on the molecular mechanism of nightshade in the treatment of colon cancer" was retracted in 2023. Reasons: original data or images not available; unreliable results or conclusions; concerns about the data; concerns about the results or conclusions.

### Colon cancer cell culture and grouping

The human colon cancer cell line SW480 was provided by the Cell Bank of the Chinese Academy of Sciences. SW480 cells were incubated by the addition of RPMI1640 medium containing 10% standard fetal bovine serum, 100 μg/mL streptomycin, and 100 U/mL penicillin medium and the incubator was set at 37°C with 5% CO_2_ [23]. Following full growth of the cells, 0.25% trypsin was used for digestion, and then the cells were collected and subcultured in 1:3. Quercetin was from Shanghai Yuanye Bio-Technology Co., Ltd., with purity ≥ 98% and CAS No. 117-39-5. Quercetin in different concentrations (20, 40, and 80 μmol/L) was employed to treat medium and taken as the experimental groups, the cisplatin (DDP) group (40 μmol/L) was used as the positive control group, and the non-quercetin group (0 μmol/L) as the negative control group.

### EdU staining

The effect of quercetin on the proliferation of SW480 cells was detected using the EdU cell proliferation kit (SolarBio, China). The third-generation SW480 cells were inoculated into 96-well plates, supplemented with 200 μL of 2 × 10^4^ cells/mL cell suspension to each well. After cell adherence to the wall was achieved, the cells were incubated synchronously in a culture medium containing 0.4% FBS for 72 h. Quercetin at different concentrations (0, 20, 40, and 80 μmol/L) and DDP (40 μmol/L) were added into each well and treated for 48 h, and then supplied with 100 μL of 50 μmol EdU for an additional incubation for 2 h. The culture medium was discarded followed by three cycles of washing with PBS, and cell fixation was performed subsequently using 4% paraformaldehyde and kept for 30 min. Three visual fields were randomly selected for observation and photographed under microscopy. The experiment was duplicated at least three times with six complex holes in each group. EdU positive cells displayed red fluorescence, and EdU labeling rate of positive cells = red fluorescent cell count/total cell count × 100% [24].

The article "Study on the molecular mechanism of nightshade in the treatment of colon cancer" was retracted in 2023. Reasons: original data or images not available; unreliable results or conclusions; concerns about the data; concerns about the results or conclusions.

### Detection of cell apoptosis by flow cytometry

SW480 cells were subcultured into 6-well plates and incubated by supplementing quercetin at 0, 20, 40, and 80 μmol/L or 40 μmol/L DDP for 12 h after cell adherence to the wall. The cells were centrifuged after digestion with trypsin to prepare single-cell suspension, subsequently washed, resuspended, labeled with annexin V-FITC and PI stained following the instructions of Annexin V-FITC/PI Apoptosis Detection Kit (20180126, Jiangsu KeyGEN Bio TECH Corp., Ltd), and upload for flow cytometry on the machine [25]. Each group had three replicates, and DMSO was used as the control group.

### TUNEL staining

After dewaxing, the paraffin sections were rinsed with PBS solution 3 times, and the sections were placed in boiled antigenic repair solution to repair antigens for 10 min. After cooling to room temperature, 100 μL proteinase K was added and performed transparency in a wet box for 20 min, rinsed with PBS, and incubated in 3% H_2_O_2_ solution for 10 min. Subsequently, 100 μL positive incubation solution was supplemented for incubation in a 37°C wet box for 30 min, dripped 50 μL labeled reaction solution, incubated in a 37°C wet box for 90 min, and then added 50 μL PI dye solution for reaction at room temperature for 5 min, and dried in an oven at 60°C. DAPI anti-fluorescence quenching agent was used to seal the sections, and images were captured using a microscope [26].

### Transwell assay

The cells were subsequently processed using quercetin at various concentrations (0, 20, 40, and 80 μmol/L) and DDP (40 μmol/L) for 48 h, digested with 0.25% trypsin, collected and centrifuged at 1200 r/min at room temperature for 3 min. The supernatant was removed. PBS was used to rinse twice to remove residual serum. Following suspension in a serum-free medium, the cells were counted using a cell counting plate. The cell concentration was diluted to 2 × 10^5^/mL with a serum-free medium. The 24-well plate was added with 800 μL 10% FBS medium and placed into a Transwell chamber (BD Company, USA) [27]. Cell suspension of each group was added with 200 μL in the upper chamber and cultured at 37°C with 5% CO_2_ for 48 h. Transwell was removed, the chamber was carefully cleaned with PBS once, and cell fixation was conducted by utilizing 70% iced ethanol solution for 1 h. The cells were stained with 0.5% crystal violet solution and placed at room temperature for 20 min. After PBS cleaning, the unmigrated cells on one side of the upper chamber were wiped off with a clean cotton ball, observed using a microscope and photographed to count the number of migrated cells.

The article "Study on the molecular mechanism of nightshade in the treatment of colon cancer" was retracted in 2023. Reasons: original data or images not available; unreliable results or conclusions; concerns about the data; concerns about the results or conclusions.

### Immunofluorescence

The SW480 cells were subcultured in a 24-well plate, the culture medium was replaced with either various concentrations of quercetin (0, 20, 40, and 80 μmol/L) or 40 μmol/L DDP for 12 h until the cell growth reached about 60%. After treatment, the culture medium was sucked out and discarded. Then the precooled methanol was supplemented to fix the cells at −20°C for 30 min. The cells were followed by three cycles of washing with PBS buffer, sealed with PBS buffer containing 5% bovine serum albumin (BSA) at room temperature for 2 h, and washed with PBS buffer three times. The primary antibody was added and incubated overnight at 4°C, and washed three times. The cells were subsequently supplemented with fluorescein isothiocyanate (FITC) labeled secondary antibody, incubated 40 min at room temperature, followed by three cycles of PBS washing and observed under a fluorescence microscope [28].

### Establishment and grouping of a nude mouse model of colon cancer tumor transplantation

SPF grade BALB/C nude mice, aged 6 weeks and weighing at 17.6 ± 2.3 g at the beginning of the experiment, were purchased from Chongqing Aissier Biological Technology Co., Ltd. The animals were raised in a sterile environment at a temperature of 26–28°C, humidity 50–60% under a 12 h light and dark cycle. The mice were supplied food and water ad libitum. The experiment was carried out after 7 days of adaptive feeding. Colon cancer SW480 cells were set at a density of 2 × 10^7^ cells/mL. Then, 0.2 mL cell suspension previously described was subcutaneously injected into the corresponding part in the neck of nude mice and the nude mouse model of tumor transplantation was established. On the following day, the model animals were randomly classified into five groups: a model group, a positive control group, low, medium, and high doses quercetin groups, 10 in each group. The low, medium, and high doses quercetin groups were administered 30, 60, and 100 mg/kg quercetin by gavage after model construction, respectively. The model group was administered an identical volume of 0.9% sodium chloride injection. The positive control group was administered with 3 mg/kg DDP by intraperitoneal injection once daily and lasted for 4 weeks by gavage. Tumorigenesis, tumor growth, and mental state of mice in each group were observed. Body weight, activity, and defecation were recorded in each group. Upon experiment completion, the mice were sacrificed and sampled by the cervical dislocation method.

The article "Study on the molecular mechanism of nightshade in the treatment of colon cancer" was retracted in 2023. Reasons: original data or images not available; unreliable results or conclusions; concerns about the data; concerns about the results or conclusions.

### Western blotting

The cells were lysed with RIPA lysate (300 μL per well) on ice for 30 min and centrifugated at 12,000 × g for 10 min after cell lysates were carefully scraped. The supernatant was collected and kept at −80°C for later use. Total protein concentration in the samples was determined using BCA method. Following the addition of SDS-PAGE loading buffer, the sample was bathed in boiling water for 10 min. Protein was isolated with 15% SDS-PAGE and then delivered to a PVDF membrane. The PVDF membrane was subsequently blocked with TBST buffer containing 5% skimmed milk at room temperature for 1 h. After sealing, corresponding primary antibodies were added and incubated overnight at 4°C. Following the PVDF membrane was rinsed using TBST three times, horseradish peroxidase-labeled secondary antibodies were incubated at room temperature for 1 h. Subsequently, the PVDF membrane had three cycles of washing with TBST buffer, and the chemiluminescence results were photographed using a GE AI600 imager [29]. The ImageJ software (NIH) was utilized for gray value analysis of each target strip. GAPDH was taken as an internal reference, the gray value ratio of the target protein to the internal reference was calculated, and the protein expression levels of each group were compared. The sources of used primary antibodies were listed below: anti-p-PI3K (A4860, abclonal), anti-p-AKT (AP0637, abclonal), anti-BAX (A15646, abclonal), anti-caspase-3 (A0214, abclonal) and anti-GAPDH (AC002, abclonal).

### Immunocoprecipitation (Co-IP) [30]

Biotin-labeled quercetin was inoculated into SW480 cell suspension and cultured for 24 h and centrifugated to collect cells. The cells were washed twice with precooled PBS, which was sucked dry at the last time. Precooled RIPA Buffer was added. The cells were scraped off the petri dish or culture flask using a precooled cell scraper, the suspension was transferred to a 1.5 EP tube and then vibrated in a horizontal shaker mildly at 4°C for 15 min. After centrifugation, a new centrifuge tube was used for supernatant transfer. Protein A agarose preparation was performed and beads were followed by two cycles of PBS washing. The concentration was set at 50% with PBS. Of each 1 mL of total protein, 100 μL Protein A agarose beads (50%) were supplemented, vibrated at 4°C for 10 min for removal of the specific heteroprotein and background reduction. Following centrifugation at 14,000 × g at 4°C for 15 min, Protein A beads were removed when the supernatant was transferred to a new centrifuge tube. A standard protein curve was plotted, and protein concentration was determined. Dilution of total protein was conducted over 10 folds before the determination to minimize the effects of detergent in the cell lysate. An addition of 500 μL total protein was supplemented to primary antibodies and slowly shook the mixture of antigen–antibody overnight at 4°C or at room temperature for 2 h. Subsequently, 100 μL Protein A agarose beads were supplied to capture antigen–antibody complexes and vibrated slowly at 4°C overnight or at room temperature for 1 h. The agarose bead antigen antibody complexes were centrifugated instantaneously at 14,000 × g for 5 s and harvested for later use. The supernatant was removed after three cycles of washing with precooled RIPA buffer. The agarose bead-antigen-antibody complexes were suspended with 60 μL 2× sample loading buffer, mixed gently, boiled for 5 min, and identified the binding proteins using Western blot analysis.

The article "Study on the molecular mechanism of nightshade in the treatment of colon cancer" was retracted in 2023. Reasons: original data or images not available; unreliable results or conclusions; concerns about the data; concerns about the results or conclusions.

### Statistical analysis

Data statistics and plotting analysis were performed using GraphPad Prism 6 software. The collected data were expressed as mean ± standard deviation (mean ± SD). Mean analysis of multiple groups was subjected to one-way ANOVA. P values < 0.05 were regarded statistically significant.

## Results

In this paper, network pharmacological analysis was performed, TCMSP and GeneCards were employed to probe the effective components, targets, and potential mechanisms of nightshade in the treatment of colon cancer, and the relationship network diagram of ‘traditional Chinese medicine – component – target – disease’ was constructed, the regulatory effect of quercetin on core targets and major signaling pathways were confirmed. EdU staining, flow cytometry, TUNEL, Western blotting, and immunofluorescence analysis were used to detect the effects of quercetin on the proliferation and apoptosis of SW480 cells, as well as the regulation of PI3K/AKT pathway. Quercetin can inhibit the expression of activated phosphorylated PI3K/AKT and up-regulate the expression of apoptotic proteins caspase-3 and BAX. Meanwhile, in vivo experiments showed that quercetin also showed significant antitumor effects on human colon cancer cells SW480 in nude mice bearing tumors. In addition, the Co-IP experiment verified that PIK3CA can directly bind to quercetin. Therefore, taken together it is considered that the mechanism of nightshade in inhibiting the activated PI3K/AKT signaling pathway through quercetin, thereby promoting the apoptosis of colon cancer cells and treating colon cancer.

### Network pharmacological analysis

In the TCMSP database, 7 principal active ingredients of nightshade were retrieved including quercetin, with 151 corresponding targets. The corresponding targets were overlapped with 484 colon cancer targets collected from the GeneCards database, and 44 overlapped targets were collected (Figure 1a). A diagram of the drug-component-target-disease network was constructed subsequently, with blue representing the overlapped targets and pink representing the active components of nightshade. Quercetin indicated the highest Degree Centrality (DC) value, suggesting that it might be essential in the treatment of colon cancer (Figure 1b). Go analysis and KEGG pathway analysis were performed on the 44 targets using ClueGo a plugin of Cytoscape to further explore the possible genes involved in treating colon cancer by nightshade administration, as well as the involved biological pathways and signaling pathways. GO analysis included 172 entries of biological process (BP), 45 entries of molecular function (MF), and 0 entries of cell component (CC) [31]. The 20 entries of the largest P values (Term) were selected for visual analysis. The GO analysis indicated the most targets enriched in BP ‘nuclear receptor activity, muscle cell proliferation, phosphatidylinositol 3-kinase signaling, ligand-activated transcription factor activity, and oxidoreductase activity’ (Figure 2a and b). Seventy-two signaling pathways were identified using KEGG pathway enrichment analysis, and the results indicated five targets with the most significant P values including PIK3R1, PIK3CA, AKT1, AKT2, and MAPK8. And the five most significant p-value signaling pathways were proteoglycans in cancer, acute myeloid leukemia, focal adhesion, VEGF signaling pathway, and pancreatic cancer (Figure 2c). Based on the above results, we selected quercetin and PI3K/Akt signaling pathway for further experiments at the cell and animal levels so that the therapeutic effect of quercetin, the main active ingredient of nightshade, on colon cancer could be verified and its molecular mechanism could be explored.

The article "Study on the molecular mechanism of nightshade in the treatment of colon cancer" was retracted in 2023. Reasons: original data or images not available; unreliable results or conclusions; concerns about the data; concerns about the results or conclusions.

**Figure 1.** Network pharmacological analysis of Long kui on colon cancer. (a) Screening of potential anti-colon cancer targets of Long kui. The corresponding targets were overlapped with 440 colon cancer targets and 44 overlapped targets were collected. (b) Network of the drug-component-target-disease. Blue represents the overlapped targets and pink represents the active components of nightshade.

**Figure 2.** Go analysis and KEGG pathway analysis. (a, (b) The top 20 GO terms of common targets. The Y axis on the left is the GO terms, and the X axis is P values. (c) The top 20 KEGG pathway of common targets. The right side is the name of the signaling pathways, and the left side is the targets. The darker the color of the inner circle on the left is, the greater the P value of the corresponding gene pathway.

### Influence of quercetin on SW480 cell growth cultured in vitro

EdU staining results indicated that red fluorescence decreased as the quercetin concentration increased, whereas positive EdU cell count decreased in a dose-dependent fashion (Figure 3a and b). Proliferation-related protein expression in SW480 cells was determined by immunofluorescence, and the findings indicated high expression of Ki67 protein [32] in SW480 cells of colon cancer tissues cultured in vitro (Figure 3c and d). Following quercetin treatment at different concentrations, the expression levels of both were decreased in a dose-dependent manner. The findings indicated that quercetin could inhibit the proliferation rate of SW480 cells in a dose-dependent manner. The TUNEL assay also indicated the role of quercetin in promoting apoptosis of SW480 cells in a dose-dependent manner when it was compared with the model group (Figure 4a). Furthermore, cell apoptosis was detected by flow cytometry. Compared with the control group, apoptosis of quercetin groups with different concentrations was markedly increased (Figure 4b).

**Figure 3.** Influence of quercetin on SW480 cell growth cultured in vitro. (a) A gradient concentration of quercetin acts on SW480 cells. Use EdU staining to mark cells in the proliferation stage, and DAPI staining to count the total number of cells. Red fluorescence represents EdU positive cells. (b, c) The quantified effect of quercetin on cell growth illustrated as bar figures with statistical analysis. (d) Immunofluorescence staining was performed on the Ki67 protein of each group of SW480 cells. Scale bar: 50 μm. The experiment had three independent repeats. Data were presented as mean ± SD (n ≥ 3 experiments). *p < 0.05, **p < 0.01, ***p < 0.001, based on one-way ANOVA, followed by Tukey’s test.

**Figure 4.** Quercetin promotes apoptosis and inhibits migration of SW480 cell. (a) TUNEL analysis of apoptosis was performed after treatments with quercetin (20, 40, and 80 μmol/L) and DDP (40 μmol/L). (b) Flow-cytometric analysis of apoptosis was performed after treatments with quercetin (20, 40, and 80 μmol/L) and DDP (40 μmol/L). (c) The pictures of adherent cells were photographed under a microscope. The invaded cells through the transwell membrane were detected by determining the area of crystal violet staining. A gradient concentration of quercetin was used to act on SW480 cells, the more quercetin concentration was, the fewer invaded cells were.

Transwell experiment results showed that the number of invaded cells was greatly reduced in each administration group compared with the control group, and the more quercetin concentration was, the fewer invaded cells were detected (Figure 4c). Quercetin could reduce the SW480 cell migration in a dose-dependent manner.

The article "Study on the molecular mechanism of nightshade in the treatment of colon cancer" was retracted in 2023. Reasons: original data or images not available; unreliable results or conclusions; concerns about the data; concerns about the results or conclusions.

### Effect of quercetin on the PI3K/Akt signaling pathway in SW480 cells

Western blot results suggested that the phosphorylation levels of PI3K and AKT were markedly decreased in the quercetin treatment group compared with the control group without quercetin treatment, and the difference between each group was statistically significant, which was positively correlated with quercetin concentrations (Figure 5a). Moreover, the expression levels of caspase-3 and BAX [33–35] were increased after quercetin treatment, suggesting that quercetin might upregulate the expressions of apoptosis-related proteins by inhibiting the PI3K/AKT pathway activation. After the biotin-labeled quercetin was incubated with the total cell protein and coprecipitation, Western blot assays discovered that PIK3CA was directly bound to quercetin, while AKT failed to indicate the binding effect (Figure 5b).

**Figure 5.** Effect of quercetin on the PI3K/Akt signaling pathway in SW480 cells. (a) The left is the protein expressions of p-Akt, p-PI3K, Bax, caspase-3 and GAPDH, which were treated as in Figure 4a and the proteins were isolated and analyzed using Western blotting. GAPDH expression served as an internal control. The right represents the bar graphs of proteins quantified using bands’ gray value by Image J. (b) Co-IP assay shows PIK3CA was directly bound to quercetin, while AKT failed to indicate the binding effect. IgG expression served as a negative control. Data were presented as mean ± SD (n ≥ 3 experiments). *p < 0.05, **p < 0.01, ***p < 0.001, based on one-way ANOVA, followed by Tukey’s test (more than two groups).

### Effect of quercetin on tumor volume and tumor inhibition rate

The addition of quercetin effectively inhibited tumor volume and weight gain of mice compared with the control group, and the inhibitory effect increased with the increase of quercetin concentration (Figure 6a). No significant difference was revealed in the inhibitory rate between the positive control group and the quercetin treatment group. Western blot analysis indicated that after quercetin treatment, the protein expressions of p-PI3K and p-AKT were decreased, whereas the expressions of caspase-3 and BAX were increased (Figure 6b). Animal experiments further showed that quercetin might inhibit the occurrence and development of colon cancer by suppressing the PI3K/Akt pathway activation and upregulating expressions of apoptosis-related proteins, thereby inhibiting the occurrence and development of colon cancer.

The article "Study on the molecular mechanism of nightshade in the treatment of colon cancer" was retracted in 2023. Reasons: original data or images not available; unreliable results or conclusions; concerns about the data; concerns about the results or conclusions.

**Figure 6.** Effect of quercetin on tumor volume and tumor inhibition rate. (a) SPF grade BALB/C nude mice were treated with 0.9% sodium chloride, DDP (3 mg/kg), and quercetin (30, 60, and 100 mg/kg) once per day and lasted for 4 weeks by gavage. The addition of quercetin effectively inhibited tumor volume and weight gain in mice. (b) The stripped tumor body was subjected to Western blot. The figures above were the protein expressions of p-Akt, p-PI3K, Bax, caspase-3, and GAPDH, which were treated as in (a) and the proteins were isolated and analyzed using Western blotting. GAPDH expression served as an internal control. Thfige below represented the bar graphs of proteins quantified using bands’ gray value after treatments as in (a). Data were presented as mean ± SD (n ≥ 3 experiments). *p < 0.05 based on one-way ANOVA, followed by Tukey’s test (more than two groups).

## Discussion

Colon cancer ranks among the top three major malignancies with high morbidity and mortality. The occurrence of this disease is correlated to multiple factors of cell proliferation, metastasis, apoptosis, tumor microenvironment, and autoimmune system. TCM therapies have been widely introduced in treating cancer, acting on diverse signal transduction pathways with few adverse reactions [36]. The traditional Chinese medicine nightshade has been reported that it can play an anti-tumor role by inhibiting cell adhesion, tumor cell infiltration and metastasis, and improving the immune function of the body [37]. Unfortunately, little has been known about the molecular mechanism of how nightshade inhibits colon cancer SW480 cells. Taken together, the present study combined the principle of holistic dialectical TCM with the characteristics of network pharmacology [38] to comprehensively investigate the anti-tumor material basis and action mechanism of nightshade. Meanwhile, it further explored the effect of quercetin, an active ingredient of nightshade, on colon cancer and its molecular mechanism in both vivo and vitro experiments.

After network pharmacological analysis, there were 7 active components screened out, and 44 overlapped action targets were all associated with colon cancer, among which quercetin had the highest DC value. The results indicated that quercetin produced a vital role in the treatment of colon cancer. Besides, KEGG pathway enrichment results indicated that PIK3R1, PIK3CA, AKT1, and AKT2 genes were of great significance in the treatment of colon cancer. Previous research has demonstrated that the PI3K/Akt signaling pathway is essential in tumor genesis, development, and radiation resistance [39]. It is involved in multiple cell activities and metabolism regulation, and it is intimately correlated with the proliferation, apoptosis, cycle regulation, angiogenesis, invasion, metastasis, and chemoradiotherapy resistance of cancer cells. Quercetin is one of the active components of the Chinese herb nightshade, featuring a wide range of pharmacological activities. It can regulate intracellular and extracellular signaling pathways related to the progression of diverse diseases, anti-inflammatory, antiviral, anti-cancer, prevention, and treatment of cardiovascular and cerebrovascular diseases [40,41]. Cell and animal experiments have demonstrated that quercetin can inhibit the expressions of p-PI3K and p-AKT in cells and tumor tissues, thereby inhibiting the activation of the PI3K/Akt signaling pathway. Apoptosis is a common form of tumor cell death, and PI3K/Akt inhibits apoptosis through various mechanisms [42]. Activation of PI3K/Akt can activate X-linked apoptosis inhibitor protein (XIAP), a member of the apoptotic inhibitor protein family, and thereby inhibiting cell apoptosis by selectively inhibiting caspase [43,44]. Additionally, activated PI3K/Akt enters the nucleus and regulates downstream proteins including mTOR, Bad, caspase-9, NF-κB, and the forkhead frame transcription factor O subfamily, thereby regulating cell survival, proliferation, apoptosis, and angiogenesis [45]. The present study indicates that the protein expressions of Bax and caspase-3 were increased after quercetin administration, suggesting that quercetin treatment could increase apoptosis of tumor cells.

The article "Study on the molecular mechanism of nightshade in the treatment of colon cancer" was retracted in 2023. Reasons: original data or images not available; unreliable results or conclusions; concerns about the data; concerns about the results or conclusions.

As cancer cells are characterized by infinite multiplication, growing studies have shown that quercetin can mediate the proliferation of cancer cells in time-dependent and concentration-dependent manner [46]. Apoptosis is known as one of the programmed cell death, the process maintains the balance of survival and death of cells. Apoptotic signals protect the integrity of the genome, but apoptotic defects may promote the occurrence of tumors [47]. Tumor cells may escape apoptosis and be capable of resistance to apoptotic factors via various molecular mechanisms [48]. Tumor therapy highlights apoptosis. The efficacy of most anticancer drugs is achieved by inducing apoptosis of their sensitive cells [49]. Quercetin can induce apoptosis of colon cancer cells in some studies [50]. This study employed flow cytometry and Tunel assays to detect changes in apoptosis of SW480 cells treated with quercetin at different concentrations, which also indicated that apoptosis increased as drug concentrations increased. Additionally, the invasiveness of tumor cells was intimately associated with the development and metastasis of cancer. In this study, migration ability of SW480 cells was also detected using Transwell assay, indicating that quercetin could inhibit the migration ability of SW480 cells in a concentration-dependent manner, which was consistent with previously described using additional methods. Taken together, the present study demonstrated that the anticancer activity of quercetin was closely related to its inhibition of proliferation and metastasis of cancer cells and induction of apoptosis. Furthermore, it has been reported that quercetin combined with chemotherapeutic agents can sensitize chemotherapy and effectively reverse the multi-drug resistance of tumor cells. This marks another mechanism of the anticancer effect utilizing quercetin.

The article "Study on the molecular mechanism of nightshade in the treatment of colon cancer" was retracted in 2023. Reasons: original data or images not available; unreliable results or conclusions; concerns about the data; concerns about the results or conclusions.

## Conclusion

The present study identifies potential active components and action targets of nightshade in treating colon cancer in a network pharmacological approach. Further in vivo and in vitro experiments indicate that quercetin mediate the phosphorylation and activation of the PI3K/Akt signaling pathway and upregulate expressions of apoptotic proteins caspase-3 and BAX, thereby inhibiting the proliferation of SW480 cells and promoting cell apoptosis. Additionally, we demonstrated the presence of a direct binding effect of quercetin and PI3K. Taken together, the mechanism of nightshade in colon cancer treatment might be the inhibitory role of quercetin in the proliferation, migration, and apoptosis promotion of colon cancer cells by mediating the PI3K/Akt-dependent signaling pathway. Meanwhile, the results of bioinformatics analysis coincide with those of previous studies, suggesting that it is reliable to figure out TCM therapeutic targets and their possible mechanisms in a bioinformatic approach.

## Highlights

1. Quercetin inhibits the proliferation and migration of colon cancer cells.
2. Quercetin could promote apoptosis of colon cancer cells in a dose-dependent manner.
3. Quercetin shows an antitumor effect on human colon cancer in nude mice.
4. PIK3CA could bind to quercetin directly.
5. Quercetin could inhibit the activation of the PIK3/AKT signaling pathway.
